# Prognostic impact of prognostic nutritional index on renal cell carcinoma: A meta-analysis of 7,629 patients

This article has been retracted.

**DOI:** 10.1371/journal.pone.0265119

**Published:** 2022-03-21

**Authors:** Qingping Peng, Ling Liu, Ting Li, Changjiang Lei, Huan Wan

**Affiliations:** 1 Department of Nephrology, The Fifth Hospital of Wuhan, Wuhan, Hubei, China; 2 Department of Stomatology, Parrot Street Community Health Service Center Affiliated of the Fifth Hospital of Wuhan, Wuhan, Hubei, China; 3 Department of General Medicine, Wulidun Neighborhood Community Health Service Center Affiliated of the Fifth Hospital of Wuhan, Wuhan, Hubei, China; 4 Department of Oncology, The Fifth Hospital of Wuhan, Wuhan, Hubei, China; 5 Department of Radiotherapy Center, The Fifth Hospital of Wuhan, Wuhan, Hubei, China; UNIBA: Universita degli Studi di Bari Aldo Moro, ITALY

## Abstract

**Background:**

Prognostic nutritional index (PNI) is a parameter which reflects nutritional and inflammatory status. The prognostic value of PNI in renal cell carcinoma (RCC) remains in debate. The aim of this study is to evaluate the prognostic value and clinicopathological features of PNI in RCC.

**Methods:**

A literature search was performed in the databases of PubMed, Embase, Web of Science, and Cochrane Library. Hazard ratios (HRs), odds ratios (ORs), and 95% confidence intervals (CIs) were extracted for meta-analysis. The association between PNI and overall survival (OS), cancer-specific survival (CSS), disease-free survival (DFS), progression-free survival (PFS), recurrence-free survival (RFS), and clinicopathological factors were evaluated.

**Results:**

Eleven studies involving 7,629 patients were included for meta-analysis. A decreased PNI was shown to be a significant predictor of worse OS (HR = 2.00, 95%CI = 1.64–2.42, p<0.001), CSS (HR = 2.54, 95%CI = 1.61–4.00, p<0.001), and DFS/PFS/RFS (HR = 2.12, 95%CI = 1.82–2.46, p<0.001) in RCC. Furthermore, a low PNI was correlated with Fuhrman grade III-IV (OR = 1.96, 95%CI = 1.27–3.02, p = 0.002), T stage T3-T4 (OR = 2.21, 95%CI = 1.27–3.87, p = 0.005), presence of sarcomatoid differentiation (OR = 5.00, 95%CI = 2.52–9.92, p<0.001), and presence of tumor necrosis (OR = 3.63, 95%CI = 2.54–5.19, p<0.001).

**Conclusion:**

PNI is an independent prognostic indicator of survival and associated with Fuhrman grade, T stage, sarcomatoid differentiation, and tumor necrosis in patients with RCC.

## Introduction

Kidney cancer is the 13th most common cancer worldwide [1]. It is estimated that there are 403,262 new cases diagnosed and 175,098 cancer-related deaths of kidney cancer in 2018 globally [2]. The most common type of kidney originating cancer is renal cell carcinoma (RCC) [1]. When initially diagnosed, bout 70% of patients with RCC have localized diseases and the remaining 30% are at regional metastatic and distant metastatic status [3]. Although most patients with RCC at localized stages are treated by surgical resection, RCC remains one of the most lethal urological malignancies [4]. Between 20% and 40% of patients with localized RCC experience disease relapse after curative intent surgery [5]. Patients with advanced RCC have a median survival of 2 years [6]. The prognostic factors play a pivotal role in identifying high-risk patients and optimizing of clinical assessment tools for patients with RCC [7].

Accumulating evidence has shown the association between prognostic nutritional index (PNI) and prognosis of various malignancies in recent years [8–12]. PNI is derived from the following formula: serum albumin (g/L) + 5 × peripheral lymphocyte count (10^9^/L), which both evaluates the nutrition and immunologic status of patients [9]. PNI was firstly reported by Buzby and colleagues [13] in 1980 and was regarded as a simply obtained nutritional and immunological parameter calculated with serum albumin level and peripheral lymphocyte count of the laboratory test. Then in 1984, Onodera et al. [14] simplified PNI and confirmed that low PNI was associated with poor prognosis after gastrointestinal surgery of malnourished cancer patients [14]. Onodera firstly introduced PNI in the prognostication of patients with cancer [14]. The prognostic significance of pretreatment PNI has been verified in many tumors including non-small cell lung cancer (NSCLC) [15], breast cancer [12], glioblastoma [16], oral squamous cell carcinoma [17], gastric cancer [18], and thyroid carcinoma [19]. The low PNI was shown as a significant prognostic factor. Previous studies have investigated the prognostic impact of PNI on RCC, with conflicting results presented [20–23]. Therefore, to clarify the prognostic role of PNI in RCC, we carried out a meta-analysis of the current published evidence on PNI and survival of RCC. In addition, we explored the association between PNI and clinical factors in PNI in this meta-analysis.

## Materials and methods

### Study guideline

We performed the current meta-analysis according to Preferred Reporting Items for Systematic Reviews and Meta-Analyses guideline [24]. Approval of an ethics committee or institutional review board is not needed because this is a meta-analysis.

### Publication search

The literature databases of PubMed, Embase, Web of Science, and Cochrane Library were retrieved. The databases were searched from inception up to June 2021. We searched the literature using the following strategies: (PNI OR prognostic nutritional index) AND (renal cell carcinoma OR RCC OR kidney cancer OR kidney neoplasms). And studies from the bibliographies of retrieved articles were also scanned for pertinent publications.

### Inclusion and exclusion criteria

We recruited eligible studies according to the following inclusion criteria: (1) the publication are English literature; (2) patients were diagnosed with RCC by histopathological or pathological analysis; (3) the PNI was measured and recorded before surgery or treatment in laboratory test; (4) survival endpoints, such as overall survival (OS), disease-free survival (DFS), progression-free survival (PFS), recurrence-free survival (RFS), and cancer-specific survival (CSS) were explored in the studies; (5) studies evaluated the prognostic clinicopathologic and value of PNI for survival endpoints and hazard ratios (HRs) with 95% confidence intervals (CIs) were provided. The exclusion criteria were as follows: (1) meeting abstracts, case reports, reviews, letters, and comments; (2) animal studies; (3) studies with overlapping patients; (4) studies with insufficient data for meta-analysis.

### Data extraction and quality evaluation

A standardized data collection form was employed to extract the following information by two authors (Q.P. and L.L.) independently: first author, year of publication, country, number of patients, sex, recruitment period, study design, metastatic status, follow-up period, clinical treatments, PNI cut‐off value, and numbers of patients with low/high PNI. In case of any discrepancies during data extraction, two investigators (C.L. and H.W.) will discuss to consensus reached. The quality of included studies was assessed by the Newcastle–Ottawa Scale (NOS) (http://www.ohri.ca/programs/clinical_epidemiology/oxford.asp). It assessed study quality by 3 classifications including selection, comparability and outcome. NOS has a full score of 9 and studies obtained more than 6 are regarded of high-quality studies.

### Statistical analysis

All statistical procedures in this meta-analysis were performed using Stata version 14.0 (Stata Corp LP, College Station, TX, USA). The prognostic value of PNI for OS, CSS, and DFS/PFS/RFS were evaluated by combined HRs and 95%CIs. If HRs and 95% CIs were not directly reported by articles, they were calculated from Kaplan–Meier curves according to Parmar’s methods [25]. The association between PNI and clinicopathological factors were assessed by pooling odds ratios (ORs) and 95%CIs. We adopted the χ2 and Higgins I^2^ to measure heterogeneity among the included studies. The results of P < 0.1 and I^2^ > 50% were considered indicative of significant heterogeneity. If no significant heterogeneity was detected, a fixed effect model was used. Otherwise, a random effect model was selected. We carried subgroup analysis to detect the source of heterogeneity. The Begg’s funnel plot and Egger’s linear regression teats were used to evaluate potential publication bias. The p<0.05 was considered as statistically significant.

## Results

### Literature search procedures

As shown in Fig 1, a total of 454 articles were retrieved after initial search of the databases. However, among them, 292 studies remained after exclusion of duplicates. Then 276 records were removed by screening title and abstract, and 16 studies were evaluated by full-text examination. After full-text reading, a total of 5 studies were eliminated for the following reasons: 3 studies did not provide sufficient data for analysis and 2 studies recruited overlapped patients. Finally, 11 studies with 7,629 patients [20–23, 26–32] were included in the meta-analysis.

**Fig 1:** Flow chart of literature search strategies.

### Characteristics of included studies

The included studies all reported association between PNI and survival outcomes, including 9 studies for OS [21–23, 26–29, 31, 32], 5 studies for CSS [20, 23, 26, 29, 30], and 8 studies for DFS/PFS/RFS [20–23, 27, 28, 30, 32]. Regarding geographical regions, 5 studies are from China [22, 23, 28, 29, 32], 3 from Korea [26, 27, 30], and one each from Austria [20], United States [21], and Turkey [31]. All included studies are of retrospective study design. Eight studies use surgery [20, 21, 23, 26, 28–30, 32] and 3 studies adopt targeted therapy [22, 27, 31] as treatment method. The cut-off values of PNI are various among included studies, ranging from 38.5 to 51.62, and the median value is 48. The included are published from 2015 to 2021, indicating the recent interest of prognostic role of PNI for RCC. The NOS scores of included studies are from 6 to 9 and are all of high quality. The detailed characteristics and quality assessment of eligible studies are shown in Table 1.

**Table 1:** Basic characteristics of included studies.

Study	Year	Country	Sample size	Sex (M/F)	Study design	Metastatic status	Treatment	Follow-up (month) median(range)	Cut-off value	No. of patients with PNI (low/high)	Survival outcomes	NOS score
Hofbauer, S. L.	2015	Austria	1344	892/452	Retrospective	Mixed	Surgery	40	48	481/863	CSS, DFS	8
Broggi, M. S.	2016	United States	341	204/115	Retrospective	Mixed	Surgery	NA	44.7	168/172	OS, RFS	7
Jeon, H. G.	2016	Korea	1437	1011/426	Retrospective	Mixed	Surgery	68.6 (1.2–212.6	51	477/960	OS, CSS	8
Cai, W.	2017	China	178	135/43	Retrospective	Metastatic	Targeted therapy	22	51.62	80/98	OS, PFS	7
Kwon, W. A.	2017	Korea	125	99/26	Retrospective	Metastatic	Targeted therapy	45.3	41	57/68	OS, PFS	8
Peng, D.	2017	China	1360	962/408	Retrospective	Mixed	Surgery	67(2–108)	47.6	382/978	OS, PFS	9
Zheng, Y. Q.	2018	China	635	400/235	Retrospective	Non- metastatic	Surgery	48.4	48	NA	OS, CSS	7
Hu, X.	2020	China	660	256/404	Retrospective	Mixed	Surgery	83	44.3	69/591	OS, CSS, PFS	7
Kim, S. J.	2020	Korea	459	307/152	Retrospective	Non- metastatic	Surgery	72(4–272)	51	164/259	CSS, RFS	7
Yasar, H. A.	2020	Turkey	396	258/138	Retrospective	Metastatic	Targeted therapy	NA	38.5	157/156	OS	6
Tang, Y.	2021	China	694	442/252	Retrospective	Non- metastatic	Surgery	60.9	49.08	267/427	OS, RFS	7

M: male, F: female, NA: not available, NOS: Newcastle-Ottawa Scale, OS: overall survival, DFS: disease-free survival, PFS: progression-free survival, RFS: recurrence-free survival, CSS: cancer-specific survival, PNI: Prognostic Nutritional Index.

### Prognostic role of PNI for RCC

All included studies investigated the prognostic role of PNI for survival in RCC. For OS, based on pooled data from 9 studies [21–23, 26–29, 31, 32], the HR and 95%CI are: HR = 2.00, 95%CI = 1.64–2.42, p<0.001, with significant heterogeneity (Fig 2). As for CSS, 5 studies [20, 23, 26, 29, 30] provide relevant data, and the pooled results are: HR = 2.54, 95%CI = 1.61–4.00, p<0.001 (Fig 3). Regarding DFS/PFS/RFS, according to data of 8 studies [20–23, 27, 29, 30, 32], the pooling data suggest that a low PNI indicates a worse DFS/PFS/RFS in RCC (HR = 2.12, 95%CI = 1.82–2.46, p<0.001), with non-significant heterogeneity (*I*^2^ = 35.9%, P = 0.142) (Fig 4). These results demonstrate that a decreased PNI is significantly associated with poorer OS, CSS, and DFS/PFS/RFS in patients with RCC. To further detect the source of heterogeneity, we performed subgroup analyses stratified by sample size, metastatic status, cut-off value, and treatment. As shown in Table 2, the results indicate that a low PNI still associates with inferior OS in all subgroups. For CSS, PNI with cut-off value ≥48 predicted worse CSS. And for DFS/PFS/RFS, a low PNI was a significant prognostic factor irrespective of sample size, cut-off value, and treatment methods.

**Fig 2:** Forest plot indicating the association between PNI and OS in renal cell carcinoma.

**Fig 3:** Forest plot indicating the association between PNI and CSS in renal cell carcinoma.

**Fig 4:** Forest plot indicating the association between PNI and DFS/PFS/RFS in renal cell carcinoma.

**Table 2:** Subgroup analysis of the meta-analysis for OS, CSS, and DFS/PFS/RFS.

Subgroup	No. of studies	HR (95%CI)	p	Effects model	Heterogeneity		
					*I*^2^(%)	P	
OS							
Total	9	2.00(1.64–2.42)	<0.001	Random	53.8		0.027
Sample size							
<500	4	2.08(1.58–2.74)	<0.001	Random	51.0		0.106
≥500	5	1.95(1.44–2.64)	<0.001	Random	62.6		0.030
Metastatic status							
Non-metastatic	2	2.86(1.60–5.11)	<0.001	Random	62.9		0.101
Metastatic	3	2.20(1.53–3.15)	<0.001	Random	64.5		0.060
Mixed	4	1.60(1.32–1.94)	<0.001	Fixed	0		0.960
Cut-off value							
<48	5	1.75(1.49–2.06)	<0.001	Fixed	0		0.980
≥48	4	2.44(1.57–3.79)	<0.001	Random	77.3		0.004
Treatment							
Surgery	6	1.90(1.47–2.45)	<0.001	Random	53.5		0.056
Targeted therapy	3	2.20(1.53–3.15)	<0.001	Random	64.5		0.060
CSS							
Total	5	2.54(1.61–4.00)	<0.001	Random	81.4		<0.001
Sample size							
<500	1	4.21(1.67–10.56)	0.002	-	-		-
≥500	4	2.36(1.43–3.90)	0.001	Random	85.3		<0.001
Metastatic status							
Non-metastatic	2	4.39(2.63–7.32)	<0.001	Fixed	0		0.914
Mixed	3	1.99(1.12–3.55)	0.019	Random	88.4		<0.001
Cut-off value							
<48	1	1.51(0.94–2.43)	0.086	-	-		-
≥48	4	2.91(1.76–4.82)	<0.001	Random	80.7		0.001
DFS/PFS/RFS							
Total	8	2.12(1.82–2.46)	<0.001	Fixed	35.9		0.142
Sample size							
<500	4	2.79(2.18–3.58)	<0.001	Fixed	0		0.750
≥500	4	1.82(1.51–2.19)	<0.001	Fixed	0		0.508
Metastatic status							
Non-metastatic	2	2.16(0.99–4.71)	0.054	Random	75.8		0.042
Metastatic	2	2.94(2.12–4.06)	<0.001	Fixed	0		0.769
Mixed	4	1.95(1.61–2.36)	<0.001	Fixed	0		0.617
Cut-off value							
<48	3	1.92(1.51–2.45)	<0.001	Fixed	18.7		0.292
≥48	5	2.24(1.86–2.70)	<0.001	Fixed	46.7		0.111
Treatment							
Surgery	6	1.94(1.64–2.29)	<0.001	Fixed	15.7		0.313
Targeted therapy	2	2.94(2.12–4.06)	<0.001	Fixed	0		0.769

OS: overall survival, DFS: disease-free survival, PFS: progression-free survival, RFS: recurrence-free survival, CSS: cancer-specific survival.

### The correlation between PNI and clinicopathological factors

We explored the association between PNI and clinicopathological features based on data derived from 5 studies [21–23, 26, 30]. As shown in Fig 5 and Table 3, the pooled results suggested that a low PNI was associated with Fuhrman grade III-IV (n = 5, OR = 1.96, 95%CI = 1.27–3.02, p = 0.002), T stage T3-T4 (n = 4, OR = 2.21, 95%CI = 1.27–3.87, p = 0.005), presence of sarcomatoid differentiation (n = 3, OR = 5.00, 95%CI = 2.52–9.92, p<0.001), and presence of tumor necrosis (n = 2, OR = 3.63, 95%CI = 2.54–5.19, p<0.001). However, there was no significant association between PNI and sex (n = 5, OR = 0.85, 95%CI = 0.65–1.12, p = 0.225) or histological type (n = 4, OR = 0.99, 95%CI = 0.60–1.61, p = 0.953) in RCC.

**Fig 5:** Forest plot of PNI with clinicopathological features in patients with renal cell carcinoma. (A) sex (male vs female); (B) Fuhrman grade (III-IV vs I-II); (C) T stage (T3-T4 vs T1-T2); (D) histology (ccRCC vs non-ccRCC); (E) sarcomatoid differentiation (yes vs no); (F) tumor necrosis (yes vs no).

**Table 3:** Results of the correlation of PNI with clinicopathologic characteristics of patients with RCC.

Clinicopathological factors	No. of studies	OR (95%CI)	p	Effects model	Heterogeneity *I*^2^(%) P	
Sex (male vs female)	5	0.85(0.65–1.12)	0.225	Random	51.1	0.085
Fuhrman grade (III-IV vs I-II)	5	1.96(1.27–3.02)	0.002	Random	81.1	<0.001
T stage (T3-T4 vs T1-T2)	4	2.21(1.27–3.87)	0.005	Random	88.3	<0.001
Histology (ccRCC vs non-ccRCC)	4	0.99(0.60–1.61)	0.953	Random	54.1	0.088
Sarcomatoid differentiation (yes vs no)	3	5.00(2.52–9.92)	<0.001	Fixed	0	0.979
Tumor necrosis (yes vs no)	2	3.63(2.54–5.19)	<0.001	Fixed	0	0.390

ccRCC: clear cell renal cell carcinoma; non-ccRCC: clear cell renal cell carcinoma: non-clear cell renal cell carcinoma.

### Publication bias

Begg’s test and Egger’s test were carried out to evaluate potential publication bias in this meta-analysis. As shown in Fig 6, there was non-significant publication bias in the present meta-analysis for OS, CSS, and DFS/PFS/RFS (all p>0.05).

**Fig 6:** Publication bias analysis of the enrolled analysis. (A) The Begg’s funnel plots for OS, p = 0.076; (B) The Egger’s test for OS, p = 0.228; (C) The Begg’s funnel plots for CSS, p = 1; (D) The Egger’s test for CSS, p = 0.821; (E) The Begg’s funnel plots for DFS/PFS/RFS, p = 0.711; (F) The Egger’s test for DFS/PFS/RFS, p = 0.257.

## Discussion

The prognostic value of PNI in patients with RCC were controversial according to previous studies [20–23, 26–32]. In the present meta-analysis including 7,629 patients, the results demonstrated that a low PNI was a significant prognostic factor for worse short-term and long-term survival outcomes in patients with RCC. The subgroup analyses confirmed the reliability of the results. In addition, we also investigated the connection between PNI and clinical factors in RCC, and the data showed that a low PNI suggested the progression and aggressively biological behaviors of the disease.

A number of studies have investigated the prognostic significance of PNI in diverse cancer types through meta-analytic methods [33–38]. A meta-analysis including 7 studies indicated that the low PNI was significantly associated with inferior prognosis of patients with biliary tract cancer and aggressive clinical factors [38]. Another recent meta-analysis showed that low PNI could be interpreted as adverse prognosis for patients with diffuse large B-cell lymphoma [39]. A meta-analysis with 6372 patients suggested that a low PNI was significantly associated with reduced survival and increased incidence of total and severe postoperative complications in patients with colorectal cancer [40]. Hu et al. showed that the PNI was a negative predictor for DFS, RFS, and PFS in patients with NSCLC in a meta-analysis [41]. A very recent meta-analysis demonstrated that a low PNI level was correlated with worse OS, PFS, and distant metastasis-free survival in patients suffering from nasopharyngeal carcinoma [42]. In the present meta-analysis, we identified the prognostic impact of PNI on survival outcomes in RCC, which was in accordance with previous findings in other types of cancer [33, 35, 38, 39, 41, 42]. Moreover, we also reported the correlation between a low PNI and various clinical features in RCC, which implied that PNI should be monitored in the management of patients.

Accumulating evidence have shown that the nutritional and immunization status are involved in the development and progress of malignancies, and therefore affect the survival outcomes [43]. On one hand, the low PNI could be caused by hypoalbuminemia and decreased lymphocyte counts. The serum albumin concentration is a reliable tool to screen nutritional status. And it is reported that a decreased pretreatment serum albumin level implies a poor prognosis for patients with RCC [44]. Malnutrition in patients with cancer is usually caused by loss of appetite and exhaustion due to tumor metabolism, which is reflected by hypoalbuminemia. In addition, the development of malignant tumor and metastases in liver could impair liver function and reduce albumin synthesis [44]. On the other hand, lymphocytes play an important in suppressing cancer cells proliferation and migration [45]. The infiltration of CD4+ T cells activates CD8+ T cells, and further induce cancer cell apoptosis. In addition, tumor-infiltrating lymphocytes (TILs) can exhibit cytotoxic activity toward cancer cells and can be applied in immunotherapy for patients with RCC [46]. Therefore, the low lymphocyte counts can result in an insufficient immunological activity and lead to worse prognosis in patients with RCC.

The recent studies also revealed the possible mechanisms between low PNI and poor prognosis in RCC. The metabolic reprogramming covers different processes such as aerobic glycolysis, fatty acid metabolism, and the utilization of tryptophan, glutamine, and arginine in RCC could be impaired because RCC is also a metabolic disease [47]. In addition, in RCC the Warburg effect is a grade-dependent feature [48], and fatty acid oxidation can be activated for different grade-dependent metabolic needs [49]. In addition, Lucarelli et al. find that oncogenic signaling pathways may promote ccRCC through rerouting the sugar metabolism. Blocking the flux through this pathway may serve as a novel therapeutic target [50]. An integrated multi‐omics characterization reveals a distinctive metabolic signature and the role of NDUFA4L2 in promoting angiogenesis, chemoresistance, and mitochondrial dysfunction in ccRCC [51]. Moreover, the subcellular distribution of phospholipid-binding protein annexin A3 in the cellular endocytic compartment suggests its involvement in modulation of vesicular trafficking, and it might serve as a putative mechanism of lipid storage regulation in ccRCC cells, opening novel translational outcomes [52]. Stearoyl-CoA desaturase (SCD1) inhibition significantly reduced cancer cell proliferation and increased cisplatin sensitivity, suggesting that this pathway can be involved in ccRCC chemotherapy resistance [53]. In addition, renal cell carcinoma is one of the most immune-infiltrated tumors [54, 55]. Emerging evidence suggests that the activation of specific metabolic pathway have a role in regulating angiogenesis and inflammatory signatures [56]. Additionally, activation of the kynurenine pathway predicts poor outcome in patients with ccRCC [57]. Features of the tumor microenvironment heavily affect disease biology and may affect responses to systemic therapy. Recent studies revealed that metabolomics represented a potential strategy for the real-time selection and monitoring of patients treated with immunotherapy in NSCLC [58].

The current meta-analysis suggested that a low PNI was predictive of poor survival outcomes of RCC, including short-term and long-term survival. In clinical practice, patients with low PNI should be managed by supplementary nutrition and be treated with other interventions which have therapeutic effect on malnutrition. Our meta-analysis suggests that PNI is an indicator for assessing survival outcomes and disease progression in RCC. Recent studies also suggested the effective prognostic role of PNI in RCC. Kwon et al. have shown that PNI is an independent prognostic factor in patients with metastatic RCC treated with targeted therapy [27]. Hu and colleagues have found that the patients of RCC with lower preoperative PNI were associated with adverse factors following nephrectomy [23]. Kim et al. have reported that The PNI is an independent prognostic factor for RFS and CSS in patients with nonmetastatic RCC treated with partial or radical nephrectomy [30].

Several limitations to our study need to be acknowledged. First of all, the included studies are all of retrospective, which may introduce selection bias. The inherent nature of retrospective studies can increase clinical heterogeneity. Secondly, the PNI cut-off values of included studies varied from 38.5 to 51.62, as a standard cut-off value of the PNI for RCC has not been determined. Thirdly, significant heterogeneity among the included studies was observed.

## Conclusion

In summary, our meta-analysis has shown that a decreased PNI is a significant prognostic factor for poorer OS, CSS, and DFS/PFS/RFS in patients with RCC. Moreover, a low PNI indicated highly aggressive biological behaviors of the disease. PNI could be applied as an independent prognostic factor for patients with RCC in clinical practice.

## Supporting information

S1 Checklist PRISMA checklist. (DOC)
